This article has been retracted.

# Effectiveness of Cognitive Behavior Therapy Combined with Eye Movement Desensitization and Reprocessing on Psychological Problems and Life Quality in Patients' Postfacial Trauma

**DOI:** 10.1155/2022/7822847

**Published:** 2022-09-07

**Authors:** Yue Lin, Wang Lv, Jun Xu, Yingying Jiang, Zheyan Chen

**Affiliations:** ^1^Department of Emergency, Wenzhou People's Hospital, Wenzhou, Zhejiang 325000, China; ^2^Department of Endoscopy Center, Wenzhou People's Hospital, Wenzhou, Zhejiang 325000, China; ^3^Department of Plastic Surgery, Wenzhou People's Hospital, Wenzhou, Zhejiang 325000, China

## Abstract

**Objective:**

To investigate the effectiveness of cognitive behavior therapy (CBT) combined with eye movement desensitization and reprocessing (EMDR) on the esteem, anxiety, depression, posttrauma stress disorder (PTSD), and posttraumatic growth in patients with facial trauma.

**Methods:**

A total of 92 facial trauma patients in Wenzhou People's Hospital from January 2017 to December 2019 were enrolled in this study. The patients were randomly divided into control group (*n* = 46) and intervention group (*n* = 46). Both of the control group and the intervention group received routine treatment, while the intervention group further received CBT combined with EMDR. Questionnaires were used to explore and record the general patient information. The Self-Esteem Scale (SES), Self-Anxiety Scale (SAS), Self-Depression Scale (SDS), Posttraumatic Stress Disorder Checklist Civilian Version (PCL-C), Posttraumatic Growth Inventory (PTGI), and World Health Organization Quality of Life-brief (WHOQOL-BREF) scores between the two groups were compared.

**Results:**

After CBT combined with EMDR intervention, the SDS and SAS scores in the intervention group were significantly decreased compared with the scores before intervention with statistically significance (*P* < 0.001). Furthermore, the PCL-C score in the intervention group showed significant decrease in comparison with the control group (*P* < 0.001), while the PTGI score in the intervention group was significantly higher than the control group (*P* < 0.001). The WHOQOL-BREF scores were increased after treatment in the two groups compared with the scores before treatment, and the scores in the intervention group were higher than those in the control group after treatment (*P* < 0.01).

**Conclusion:**

Psychological intervention therapy can effectively alleviate the anxiety, depression, and PTSD and improve the life quality and the recovery of facial trauma patients.

## 1. Introduction

Facial trauma as sign of injuries is a major challenge in public health in relation to the self-perception and self-esteem of patients [1]. Increasing evidence from psychology, anthropology, and socioeconomics has demonstrated that people with attractive facial appearance have an advantage in their social life [2–4]. Patients postfacial trauma usually receive negative social response during social interactions, leading to detrimental effects on their mental state such as depression, anxiety, and posttraumatic stress disorder (PTSD) [5, 6]. However, patients can also positively change their perspectives and undergo personal growth after a major life crisis or traumatic event [7], and this process is called posttraumatic growth (PTG). The psychological factors in the treatment of facial trauma should be paid more attention.

The PTSD treatment includes the psychological and pharmacological methods. For psychological treatment, there are trauma-focused psychological interventions such as exposure therapy and cognitive therapy and non-trauma-focused psychological interventions such as relaxation, stress inoculation training, and interpersonal therapy [8]. Eye movement desensitization and reprocessing (EMDR) and cognitive behavioral therapy (CBT) are known as the trauma-focused psychological therapies. EMDR heals people from the emotional distress [9, 10] and is prevalently applied in the treatment of PTSD patients. It mainly consists of eight phases, including recalling an image, thought, emotion, and a bodily sensation related to the traumatic event, receiving bilateral stimulation such as taps, tones, or eye movements [11]. It has been reported that EMDR is effective treatment for psychopathology and psychological problems in patients with facial trauma, which helps them to desensitize discomfort caused by traumatic experiences and reprocess them in the individual's autobiographical memory, thus achieving the goal of relieving symptoms [12]. CBT is a trauma-focused psychotherapy whose effect has been demonstrated in multiple randomized controlled trials [13–15]. Currently, CBT is also regarded as a well-established intervention to treat posttraumatic stress and related symptoms [8, 16]. The World Health Organization has recommended CBT as a treatment option for posttraumatic stress with a focus on trauma [17].

In China, the psychological intervention of posttrauma patients is not widely available. Our study is aimed at exploring the effectiveness of CBT combined with EMDR for the psychological intervention of patients with facial trauma. The findings of our study may provide evidence for the clinical effect of CBT combined with EMDR.

## 2. Materials and Methods

### 2.1. Study Participants

By convenient sampling, 92 facial trauma patients in Wenzhou People's Hospital from January 2017 to December 2019 were selected for this study. Inclusion criteria are as follows: (1) participants were educated and could read and comprehend the content of questionnaires, (2) aged between 18 and 60, (3) patients are hospitalized with facial trauma without organic brain injury and did not require craniocerebral surgery, (4) no other life-threatening or disabling injuries, (5) clear in language expression and stable in disease condition, and (6) never received CBT or EMDR interventions. Exclusion criteria are as follows: (1) patients with history of depression, anxiety disorder, or schizophrenia; (2) patients experienced death of relatives or friends or great property loss in the trauma; (3) patients complicated with other physical diseases during the treatment; and (4) patients out of contact in the follow-up or refused to accept psychological intervention or scale evaluation. Body mass index (BMI) was measured using the formula: body mass (kg)/height squared (m^2^). Significant difference between the two groups was found in the drinking history (*P* < 0.05), average length of hospital stay (*P* < 0.001), and hospitalization expenses (*P* < 0.05). There was no statistical difference in other baseline characteristics such as age, BMI, gender, and education level (*P* > 0.05). Our study was under the approval of the Ethics Committee of the Wenzhou People's Hospital, and all participants have signed the informed consent.

### 2.2. Methods

92 patients with 49 males and 43 females were randomly divided into the control group and intervention group with 46 participants in each group. Patients in the control group received routine treatment, including the posttrauma treatment, condition monitoring, health education, diet guidance, medication guidance, regular ward rounds, rehabilitation nursing, and prevention of infection and other complications. Patients in the intervention group received CBT combined with EMDR based on the routine treatment procedures. The intervention duration was once every two days from hospitalization, 60-90 minutes each time. After discharge from hospital, patients were transferred to the psychological department for further treatment or home visit. The end of treatment was determined by the condition of patients and the joint agreement of therapists and patients. The explicit procedures were as follows: (1) psychological intervention team was established, including 2 physicians, 2 nurses in charge, and 3 follow-up therapists. All the staff had years of experience in diagnosis and treatment or nursing and received professional psychological training. There were 3 national second-level psychological consultants with years of experience in clinical CBT and EMDR operation; (2) CBT operation procedures [18], in trauma-focused CBT, besides the psychological education and anxiety management (such as muscle relaxation or breathing training), exposure (body and imagined), and cognitive reconstruction (check and challenge the idea of dysfunction) are the most critical factor. Complete treatment process included 12 times of interventions. The first intervention was the narrative memories of traumatic events, and patients described the event for multiple times (≥2 times). The second intervention included the interpretation of the treatment plan, the relaxation exercise and the trauma-focused psychological education, and the introduction of the following exposure practice. The third intervention included the practice of recalling the traumatic event, exposure, and homework, The fourth to ninth intervention included homework, the relaxation exercise, psychological education, strategy management, thought intrusion, thought prevention, etc. The tenth to twelfth interventions included systematic desensitization, evaluation of stress situation grade, and scale score; (3) EMDR operation [19], first, the consultant determined the most disturbing memories about the trauma event from patients, the related negative thoughts, disturbing emotions, and positions of the patients. Then, the patients were asked to focus on the traumatic event and simultaneously followed the bilateral finger movements of counselor for about 30 seconds. After exercises, patients were asked to share any emotions/flashbacks/perceptions they noticed in the process of visual stimulation. When the patient exhibited no more emotional outbursts or any other feelings associated with the target memory, the counselor evaluated the ability of patients of detailed description until the patients could think of the trauma without disturbing emotion or physical responses. Then, we chose other targets and repeated the same procedure (trauma identification, visual stimulation, and assessment). EMDR treatment ended when the patient was able to face the reformulated goals in the imagined future scenario without emotional discomfort. The hospital stay length and treatment expense of the two groups were recorded.

### 2.3. Measures

The observation indicators were collected using questionnaires: (1) Self-Esteem Scale (SES), compiled by Rosenberg in 1965 with a total score of 40 [20]. The higher the score, the higher the self-esteem; (2) Self-Rating Anxiety Scale (SAS) and Self-Rating Depression Scale (SDS), compiled by W.K. Zung in 1965 and 1971 with a total score of 100. In the SAS, a higher score indicates a higher degree of anxiety: a score of 50-70 out of 100 suggests mild anxiety, 71-90 suggests moderate anxiety, and higher than 90 suggests severe anxiety. In the SDS, a higher score reflects a higher degree of depression: a score from 50 to 70 out of 100 represents mild depression, from 71 to 90 represents moderate depression, and higher than 90 represents severe depression; (3) PTSD Checklist-Civilian version (PCL-C) is used to evaluate the severity of PTSD symptoms. The intensity and frequency of PTSD symptoms were divided into five grades, and the higher the scores, the severer the PTSD symptoms. A total score of 38 to 49 was defined as a degree of PTSD, and those of 50 to 85 were diagnosed as PTSD. (4) Posttraumatic Growth Inventory (PTGI), compiled by Tedeschi et al., was used to assess the perceived degree of positive life change after traumatic events. It includes 21 items and explores 6 dimensions. The Likert 6-level scoring method is adopted with a total score of 105, and the higher the score, the more the posttraumatic growth. (5) World Health Organization Quality of Life-brief (WHOQOL-BREF) [21] includes a generic facet (overall quality of life and general health) and 4 domains such as physical health, psychological health, social relationships, and environment. The higher the scores, the better the quality of life. After the two groups of patients were admitted to the hospital and in stable condition, these scales were filled out under the guidance of the nurse in charge. Patients with writing ability filled out the scales by themselves, and those without writing ability were guided by the nurse. The questionnaires would be collected and checked once the patients finished. The SES, SAS, SDS, PCL-C, PTGI, and WHOQOL-BREF scales were also filled out by patients in the intervention group after the intervention period and patients in the control group in the follow-up after 15-30 days discharged of hospital.

### 2.4. Statistical Analysis

SPSS 21.0 was used to perform statistical analysis. The data were expressed as the number, percent, and mean ± SD. Paired *t*-test was used for univariate analysis before and after intervention, and Student's *t*-test was used for comparison between two groups. Chi-square (*χ*^2^) test was used to assess the relationship between two categorical variables. The multivariate analysis was conducted with logistic regression analysis. *P* < 0.05 was considered statistically significant.

## 3. Results

### 3.1. Clinical Characteristics of Patients

A total of 92 cases with facial trauma were enrolled in this study. There were no statistical difference between the age, BMI, gender, place of residence, smoking history, marital history, record of children, career, education level, family monthly income, the forms of injury, treatment, complicated injury, and predicted prognosis between the intervention group and control group (*P* > 0.05). We also found the statistical difference in the drinking history (*P* < 0.05), length of hospital stay (*P* < 0.001), and treatment expenses between the two groups (*P* < 0.05), as shown in Table 1.

### 3.2. The Effect of Psychological Intervention on the Self-Esteem, Depression, and Anxiety of Patients

The effects of psychological intervention on the SES, SDS, and SAS scores before and after intervention are presented in Table 2. There was no significant difference in the SES score between the two groups before and after intervention (*P* > 0.05), but there were significant differences in SDS and SAS scores between the two groups before and after intervention (*P* < 0.001). A total of 43 patients (46.94%) in the two groups showed low self-esteem (SES < 20), 72 patients (78.26%) showed mild or more depression symptoms (SDS > 53), and 86 patients (93.48%) showed mild or more anxiety (SAS > 50).

During the follow-up period, there were 23 cases (25.00%) showed low self-esteem, 36 cases (39.13%) showed depression, and 44 cases (47.83%) showed anxiety in the control group. In the intervention group, there were 20 cases (21.74%) of low self-esteem, 9 cases (9.78%) of depression, and 19 cases (20.65%) of anxiety, respectively. The incidence of depression and anxiety was significantly different between the two groups (*P* < 0.05). The scores of depression and anxiety reduced significantly after intervention (*P* < 0.05), while the SES scores were not significantly affected. According to multivariate analysis, the SAS and SDS scores in the intervention group were significantly reduced compared with the control group (*P* < 0.05).

### 3.3. The Influence of Psychological Intervention on the PTSD and PTG of Patients

The effects of psychological intervention on PCL-C and PTGI scores are exhibited in Table 2. During the follow-up period after discharge from the hospital, 42 patients (91.30%) in the control group developed a certain degree of PTSD (PCL‐C > 38), and 22 cases (47.83%) of them were diagnosed of PTSD (PCL‐C > 50). For the intervention group, there were 15 patients (32.61%) developed a certain degree of PTSD (PCL‐C > 38), among whom 6 cases (13.04%) were diagnosed of PTSD. Both univariate and multivariate analyses demonstrated lower total PCL-C scores and higher PTGI scores in the intervention group in comparison with the control group after intervention, with statistical differences (*P* < 0.001).

### 3.4. Comparison of the Treatment Outcome between the Two Groups on the Quality of Life

The WHOQOL-BREF scores of the two groups were also compared. The results indicated that the WHOQOL-BREF scores were both increased in two groups before and after the treatment. Moreover, after the treatment, the patients in the intervention group showed higher WHOQOL-BREF scores than those in the control group, especially in the psychological health and social relationship fields (*P* < 0.01), which indicated the effect of CBT combined with EMDR on the improvement of life quality of patients with facial trauma, as shown in Table 3.

## 4. Discussion

The human face, characterized by the uniqueness, is a dynamic tool carrying information in social communication [22]. It is closely related to the sense of self, self-esteem, and identity [23, 24]. Patients with facial trauma due to violence, road accidents, burn injury, sports injuries, etc., often experience a variety of symptoms of emotional stress, including depression, anxiety, social phobia, low self-esteem, and frustration, resulting in susceptibility to psychological problems and poor life quality [25–27]. According to clinical researches, about 20%-30% patients with facial trauma show the symptoms and signs of anxiety [28, 29]. Moreover, patients with facial trauma showed increased PTSD incidence compared with the general population [30, 31]. In our study, we found that patients with facial trauma exhibited evident short-term symptoms of depression and anxiety. There were 78.26% of the patients with different degrees of depression and 93.48% of the patients of anxiety symptoms. In the follow-up periods, part of the control group patients could calm down by themselves, while there were still 39.13% of patients of depression and 47.83% of patients of anxiety to different degrees. The incidence of depression and anxiety was significantly different between the two groups (*P* < 0.05). The scores of depression and anxiety reduced significantly after intervention (*P* < 0.05), while the SES scores were not significantly affected. According to multivariate analysis, the SAS and SDS scores in the intervention group were significantly reduced compared with the control group (*P* < 0.05). Additionally, 47.83% of the patients presented the symptoms of PTSD. Therefore, patients with facial trauma are prone to adverse psychological emotions, and more attention should be paid to improving their mental health.

The management of psychological intervention of patients with facial trauma is still challenging. The EMDR and CBT are evidence-based treatment options for patients with PTSD [32]. Previous studies have compared the effect of EMDR and CBT for different mental disorders such as PTSD, obsessive-compulsive disorder, and panic disorder [33–35]. Both the two methods showed significant effect to alleviate the depression, anxiety, and behavior problems [36]. In our study, we provided CBT and EMDR interventions to patients from admission to hospital in stable condition to the follow-up home visit. After treatment, patients in the intervention group presented lower SDS, SAS, and PCL-C scores compared with the control group in the follow-up periods (*P* < 0.001). There were 9.78% patients presented depression, 20.65% presented anxiety, and 13.04% presented PTSD in the intervention group. After treatment, the PTGI score of the intervention group was significantly higher than those of the control group (*P* < 0.001). The hospital stay (*P* < 0.001) and hospital expenses (*P* < 0.05) in the intervention group were significantly lower than the control group. Moreover, compared with the control group, patients in the intervention group showed improved physical health, psychological health, social relationship, and environment (*P* < 0.01). CBT combined with EMDR intervention was effective to improve the life quality of patients with facial trauma. Therefore, based on the trusted doctor-patient relationship, doctors should actively listen to the feelings of patients and adopt the CBT combined with EMDR to affect the negative thought of patients, promoting the establishment of right cognition and recovery from trauma.

In conclusion, based on the CBT combined with EMDR psychological intervention to the patients with facial trauma, we found that psychological intervention is effective to attenuate the depression, anxiety, and PTSD and improve the posttrauma growth self-esteem as well as life quality of patients with facial trauma. The finding of our study indicates the potential of CBT combined with EMDR in the psychological intervention of facial trauma patients in clinical practice.

## Figures and Tables

**Table 1:** Demographic and baseline characteristics of the two groups.

Factors	Control group (*n* = 46)	Intervention group (*n* = 46)	*T*/*χ*^2^	*P*
Age (years)	28.70 ± 4.62	30.43 ± 5.47	1.64	0.10
BMI (kg/m^2^)	20.79 ± 2.88	20.11 ± 2.66	1.17	0.24
Gender				
Male	25 (54.35)	24 (52.17)	0.04	0.83
Female	21 (45.65)	22 (47.83)		
Residence place				
Urban	43 (93.48)	43 (93.48)	0	1
Rural	3 (6.52)	3 (6.52)		
Smoking history				
No	36 (78.26)	34 (73.91)	0.24	0.63
Yes	10 (21.74)	12 (26.09)		
Drinking history				
No	28 (60.87)	41 (89.13)	9.8	<0.05
Yes	18 (39.13)	5 (10.87)		
Marital status				
Unmarried	11 (23.91)	21 (45.65)	5.27	0.07
Married	32 (69.57)	24 (52.17)		
Divorced	3 (6.52)	1 (2.17)		
Child				
No	24 (52.17)	25 (54.35)	0.04	0.83
Yes	22 (47.83)	21 (45.65)		
Career				
Farmer/migrant worker	10 (21.74)	7 (15.22)	1.99	0.57
Enterprises and public institutions	18 (39.13)	20 (43.48)		
Others	10 (21.74)	14 (30.43)		
Jobless	8 (17.39)	5 (10.87)		
Education level				
Junior-senior high school and below	15 (32.61)	10 (21.74)	2.55	0.28
College degree/bachelor and above	30 (65.22)	36 (78.26)		
Others	1 (2.17)	0 (0)		
Family monthly income				
<5000	6 (13.04)	10 (21.74)	1.21	0.27
≥5000	40 (86.96)	36 (78.26)		
Forms of injury				
Violence	8 (17.39)	7 (15.22)	1.13	0.77
Road accident	13 (28.26)	10 (21.74)		
Fall down	19 (41.3)	24 (52.17)		
Others	6 (13.04)	5 (10.87)		
Treatment				
Conservative treatment	32 (69.57)	36 (78.26)	0.9	0.34
Surgery	14 (30.43)	10 (21.74)		
Complicated injury				
No	29 (63.04)	28 (60.87)	0.05	0.83
Yes	17 (36.96)	18 (39.13)		
Predicted prognosis				
Favorable	34 (73.91)	37 (80.43)	0.56	0.46
Poor	12 (26.09)	9 (19.57)		
Hospital stay (days)	4.94 ± 1.73	3.07 ± 0.68	6.82	<0.001
Expenses (thousand yuan)	6.37 ± 3.08	5.11 ± 2.61	2.12	<0.05

**Table 2:** Comparison of treatment outcomes between the two groups.

Indicators	Evaluation period	Control group (*n* = 46)	Intervention group (*n* = 46)	*T*	*P*	*B*	^∗^ *P*
SES score	Before intervention	19.39 ± 4.71	19.54 ± 5.21	0.15	0.88	-0.65	0.49
	After intervention	20.76 ± 3.55	19.54 ± 5.21	0.22	0.83		
SDS score	Before intervention	63.39 ± 11.71	62.24 ± 7.90	0.55	0.58	-12.97	<0.001
	After intervention	59.98 ± 9.43	46.07 ± 7.10	8.00	<0.001		
SAS score	Before intervention	64.41 ± 10.13	65.43 ± 9.73	0.49	0.62	-14.99	<0.001
	After intervention	61.5 ± 6.40	46.09 ± 11.95	7.71	<0.001		
PCL-C score	After intervention	50.00 ± 7.87	22.85 ± 13.77	7.33	<0.001	-16.05	<0.001
PTGI score	After intervention	42.24 ± 6.18	52.17 ± 10.30	5.61	<0.001	10.40	<0.001

^∗^ *P* indicates the logistic regression *P* value.

**Table 3:** Comparison of the WHOQOL-BREF indicator between the two groups.

Indicator	Control group (*n* = 46)		Intervention group (*n* = 46)		*F*
	Before treatment	After treatment	Before treatment	After treatment	
Physical health	20.6 ± 4.0	22.2 ± 3.8	20.5 ± 3.6	23.8 ± 4.2	1.94
Psychological health	17.8 ± 3.8	19.3 ± 4.1	18.2 ± 3.6	20.7 ± 3.8	2.05^∗∗^
Social relationships	8.7 ± 2.5	9.4 ± 3.2	8.9 ± 2.3	9.7 ± 2.6	6.37^∗∗^
Environment	25.9 ± 4.2	27.2 ± 4.5	26.7 ± 4.6	29.4 ± 4.1	7.53

^∗∗^ *P* < 0.01.

## Data Availability

Data generated in this study are available from the corresponding author under reasonable requests.
